# The Curative Effect of Shuangshen Decoction Combined with Immunological Preparations in the Treatment of Pediatric Nephrotic Syndrome and Its Influence on the Rate of Complicated Infection and Recurrence

This article has been retracted.

**DOI:** 10.1155/2022/3355462

**Published:** 2022-01-27

**Authors:** Naiqin Han, Jialing Xie, Qiuying Li, Haixia Li, Xiuzhen Wang, Ying Sheng

**Affiliations:** ^1^Department of Pediatric, Zhangqiu District People's Hospital, Jinan 250200, Shandong Province, China; ^2^Department of Pharmacy, Zhangqiu District People's Hospital, Jinan 250200, Shandong Province, China; ^3^Department of Imaging, Zhangqiu District People's Hospital, Jinan 250200, Shandong Province, China; ^4^Operation Room, Zhangqiu District People's Hospital, Jinan 250200, Shandong Province, China; ^5^Department of Nutriology, Zhangqiu District People's Hospital, Jinan 250200, Shandong Province, China; ^6^Department of Pediatric, The Third People's Hospital of Qingdao, Qingdao 266041, Shandong Province, China

## Abstract

**Background:**

To explore the curative effect of Shuangshen Decoction combined with immunological preparations in the treatment of pediatric nephrotic syndrome and its influence on concurrent infection and recurrence rate.

**Methods:**

Ninety children with nephrotic syndrome were divided into the routine group and the combined group. The routine group received conventional treatment and immune agents, and the combined group was treated with Shuangshen Decoction on the basis of the routine group. The clinical indexes of the two groups were analyzed and followed up. The infection rate and recurrence rate were calculated.

**Results:**

The TCM syndrome scores in the combined group were significantly lower than those in the routine group. The total effective rate of the combined group was significantly higher than that of the routine group. The recurrence rate and infection rate of the combined group were significantly lower than those of the routine group. The incidence of adverse reactions in the combined group was significantly lower than that in the routine group.

**Conclusion:**

Shuangshen Decoction combined with immune preparations is effective in treating pediatric nephrotic syndrome and can reduce the incidence of adverse reactions, infection rate, and recurrence rate.

## 1. Introduction

Pediatric nephrotic syndrome is a common pediatric kidney disease in the clinic, which mainly manifests as massive proteinuria, hypoalbuminemia, severe edema, and hypercholesterolemia [1]. Prednisone should be used as soon as possible after the diagnosis of newly diagnosed children. Relapse patients need to adjust the dose and course of treatment of glucocorticoids [2]. However, children who frequently relapse and receive long-term high-dose glucocorticoid therapy are prone to slow growth and delayed development [3]. Therefore, clinical treatment of primary nephropathy in children is based on strengthening the spleen and kidney and controlling the side effects of Western medicine as the main principles [4]. In the treatment of children with nephrotic syndrome, especially those who have not used hormones, corn silk, plantain, Lysimachia, and Pianch are commonly used [5]. Chinese medicine adjuvant therapy can alleviate the feedback inhibition effect of exogenous corticosteroids on adrenal cortex function [6]. Therefore, a comprehensive treatment plan combining traditional Chinese and Western medicine should be investigated for pediatric nephrotic syndrome.

According to the clinical manifestations of nephrotic syndrome, the traditional Chinese medicine (TCM) theory classifies it as the “edema category,” mostly yin water. Weakness of the kidney, spleen, and lung is the main cause of nephrotic syndrome, which is mainly manifested as spleen and kidney deficiency [7]. Shuangshen Decoction contains a variety of herbs. Among them, Morus mulberry can dispel rheumatism, invigorate the liver and kidney, and strengthen muscles and bones [8]. Corn silk can clear the liver, promote choleretics, diuresis, and reduce swelling. The keel can condense sweat, consolidate essence, and calm and soothe the nerves. Magnets can calm the nerves, calm the liver, and suppress the yang [9]. Polygonum multiflorum can moisten the intestines, help defecate and nourish the body. Ligusticum chuanxiong can promote blood circulation, relieve pain, and expel wind and dampness [10]. Epimedium can replenish life, nourish vital energy, strengthen muscles and bones, and nourish the kidney. Eucommia can nourish the liver and kidney and strengthen bones and muscles [11]. However, there are few relevant research reports about the use of Shuangshen Decoction in the treatment of pediatric nephrotic syndrome.

Immunosuppressants are mainly used for patients with frequent relapses of nephrotic syndrome, glucocorticoid dependence, drug resistance, or severe side effects [12]. In small doses of glucocorticoids used every other day, immunosuppressive agents can be used at the same time. Currently, commonly used clinical immunosuppressants are cyclosporine A, tacrolimus (FK506), mycophenolate mofetil, and leflunomide [13]. The dual inhibitory effect of tacrolimus makes it not only able to prevent the occurrence of immunity but also have a good therapeutic effect on the immune response and autoimmune diseases that have appeared [14]. It has been reported that the efficacy of Chinese medicine combined with immune preparations in the treatment of pediatric nephrotic syndrome is significantly higher than that of Western medicine alone [15]. The combination of Chinese and Western medicine not only expands the treatment options but also has better curative effects. Based on this, this study will explore the efficacy of Shuangshen Decoction combined with immune preparations in the treatment of pediatric nephrotic syndrome and its influence on the rate of complicated infection and recurrence in children.

## 2. Materials and methods

### 2.1. Case Grouping

90 children with nephrotic syndrome (2018.06-2021.06) admitted to the Zhangqiu District People's Hospital were selected for a retrospective study. Forty-five children who received conventional treatment and immune preparations were set as the routine group. On the basis of the conventional group, 45 children treated with Shuangshen Decoction were included in the combined group. The study was approved by the Ethics Committee of the Zhangqiu District People's Hospital (2018-086).

### 2.2. Inclusion Criteria

1. It meets the diagnostic criteria of the “Guidelines for the Diagnosis and Treatment of Common Kidney Diseases in Children (1)” [16]. The child has obvious symptoms of edema with the 24-hour urine protein quantitative ≥50 mg·(kg·24 h)^−1^, serum albumin (ALB) ≤25 g·L^−1^, and hypercholesterolemia (>5.7 mmol·L^−1^).
2. According to the “Practical Pediatrics of Traditional Chinese Medicine” [17], the child presented with syndrome of deficiency of both the lung and spleen and syndrome of spleen deficiency and dampness
3. It meets the indications for immune preparations. Immunosuppressive agents are mainly used in patients with frequent relapses of nephrotic syndrome, glucocorticoid dependence, drug resistance, or severe side effects
4. The family members of the patient agreed to this study

### 2.3. Exclusion Criteria

1. Combined with Henoch-Schonlein purpura nephritis, lupus nephritis, hereditary nephropathy, and hepatitis B-related nephritis
2. Urinary red blood cells >10/HP
3. Taking Chinese medicine for the past month
4. Combined with renal insufficiency

### 2.4. Treatment

*Routine group*: (1) Basic treatment measures were used to avoid infection and fatigue in children. Children's daily diet should be careful to avoid spicy, greasy, and irritating food. Salt should be limited during the edema period. (2) Symptomatic treatment measures. Appropriate diuretic drugs should be given, such as HMG-CoA reductase inhibitors or sodium alginate diester. Heparin anticoagulation therapy is given. Infected children need to choose antibiotics for anti-infective treatment [18–20]. (3) Tacrolimus capsule (specification: 1 mg; manufacturer: Sinopharm Chuankang Pharmaceutical Co., Ltd.; Sinopharm Zhunzi H20083943) immune preparation treatment. The first medication is 0.05-0.1 mg/kg on an empty stomach (12 h/time). The blood concentration of tacrolimus was rechecked one week later. According to the blood concentration and the condition of the child, the dosage was adjusted appropriately to maintain the blood concentration of 5-10 *μ*g/L. The treatment cycle is 1 year.

*Combined group*: Shuangshen Decoction was added on the basis of the routine group. Shuangshen Decoction prescription: 30 g Morus alba, 30 g corn silk, 30 g raw keel (first decoction), 30 g magnet (first decoction), 24 g Polygonum multiflorum, 9 g Chuanxiong, 9 g Epimedium, and 9 g Eucommia. *Decoction method*: One dose of the medicine was put into a sand jar, and cold water was added to the surface. After soaking for 30 minutes, the medicine was heated to boiling water. Then, the medicine was cooked for 25 minutes on medium-low heat. The residue was filtered to get the juice. About 100-150 mL is the first medicine. Boiled water was added to 1 finger higher than the noodles. After the water boils, the medicine was cooked for 30 minutes. Then, the residue was filtered to get the juice, about 200 mL. After mixing the first and second medicines, the medicine juice was taken in three warm doses, one dose per day. >12-year-old children need 100-120 mL/time, 3 times a day. Children aged 7-12 need 80-100 mL/time, 3 times a day. 3-6-year-old children need 50-80 mL/time, 3 times a day. The medicine juice should be taken half an hour before or after a meal.

### 2.5. Observation Index

The patient's age, course of disease, gender, body mass index (BMI), disease progression, white blood cell count, cholesterol, triglycerides, and other general information were recorded. The patient's albumin (ALB) level was detected by immunoassay. And the patient's 24 h urine protein quantitative level was recorded. According to the severity of the primary and secondary symptoms, the patient's TCM syndrome score was evaluated. The specific information about the TCM syndrome score was shown in Table 1.

The clinical efficacy of patients was evaluated according to the “Standards for Diagnosis and Efficacy of TCM Diseases and Syndromes” [21] and changes in clinical signs, 24 h urine protein quantification, and recovery of ALB indicators. Significantly effective means the obvious improvement of TCM symptoms and clinical signs and 24 h urine protein quantification ≤ 1.0 g, ALB ≥ 35 g/L. Effective means that TCM symptoms and clinical signs have improved, and 1.0g < 24 h urine protein ≤ 3.0 g, 30 g/L ≤ ALB < 35 g/L. Invalid means that TCM symptoms and clinical signs have not improved or worsened, and 24 h urine protein quantitative > 3.0 g and ALB < 30 g/L. The total effective rate of treatment = (significantly effective + effective)/total × 100%.

The occurrence of infections and adverse reactions during the treatment of patients was recorded. The types of infections mainly include upper respiratory tract infections, lower respiratory tract infections, urinary tract infections, and gastrointestinal infections. The patients were followed up for no less than 6 months to review the patient's recurrence.

### 2.6. Statistical Analysis

SPSS22.0 Software was used to calculate the differences between groups. The figure was drawn using GraphPad Prism 7 (GraphPad Software, San Diego, USA). Research data includes counts and measurements, expressed in the form of [*n* (%)] and mean ± standard deviation (SD), respectively. Chi-squared test and Student *t* test were used for difference analysis. *P* < 0.05 indicates that there is a statistical difference between the groups.

## 3. Results

### 3.1. Comparison of General Information

There was no statistically significant difference in general information between the routine group and the combined group (*P* > 0.05, Table 2). Therefore, a controlled study can be conducted.

### 3.2. Comparison of Serum Albumin and 24 h Urine Protein

The ALB level of the two groups was significantly increased after treatment. However, the ALB level of the combined group was increased significantly after 1 and 3 months of treatment compared with the routine group (*P* < 0.05, Figure 1). The 24 h urine protein quantification after treatment in the two groups was significantly decreased. However, the 24 h urine protein quantification after 1-month and 3-month treatment in the combined group was significantly lower than that in the routine group (*P* < 0.05, Figure 2).

### 3.3. Comparison of TCM Syndrome Points

The scores of TCM syndromes in the combined group were significantly lower than those in the routine group after treatment (*P* < 0.05, Table 3). The difference is statistically significant.

### 3.4. Comparison of Clinical Efficacy

The total effective rate of the combined group was significantly higher than that of the routine group (*P* < 0.05, Table 4). The difference between the groups was statistically significant.

### 3.5. Comparison of Infection Rate and Recurrence Rate

The recurrence rate and infection rate of patients in the combined group were significantly lower than those in the routine group (*P* < 0.05, Figure 3). The incidence of adverse reactions such as nausea and vomiting, acne, hypertension, and coagulopathy in the combined group was significantly lower than that in the routine group (*P* < 0.05, Table 5).

## 4. Discussion

Pediatric nephritic syndrome is second only to acute nephritis in childhood nephropathy. Conventional treatment drugs are mostly glucocorticoids and cytotoxic drugs. The short-term curative effect is remarkable. However, the long-term application of the drug has serious adverse reactions, which can easily cause symptoms such as infection, growth inhibition, water and sodium retention, and central obesity. These adverse reactions can cause the recurrence of pediatric nephritic syndrome, and it is difficult to completely cure [22]. In this study, we found that the ALB levels of the two groups after treatment were significantly increased. However, the increase in the ALB level of the combined group after 1 month and 3 months of treatment was significantly higher than that of the routine group. The 24 h urine protein quantification of the two groups was decreased significantly after treatment. However, the 24 h urine protein quantification after 1-month and 3-month treatment in the combined group was significantly lower than that in the routine group. Xu et al. also reported similar results [23]. These findings indicate that Shuangshen Decoction combined with immune preparations have a more obvious regulatory effect on the quantitative level of ALB and 24 h urine protein in children. Therefore, Shuangshen Decoction combined with immune preparations is conducive to disease control and guiding prognosis.

The scores of TCM syndromes after treatment in the combined group were significantly lower than those in the routine group. Traditional Chinese medicine believes that children's nephrotic syndrome is mostly caused by edema, proteinuria, and other symptoms. Lungs dominate qi, and poor qi movement can cause edema. The spleen is the source of biochemistry, and it is a syndrome of phlegm and dampness block caused by the failure of the spleen [24]. The kidney is a visceral organ with water, and the lack of kidney qi causes abnormal urination or edema. Therefore, the main treatment is to warm the spleen and kidney, promote blood circulation to remove stasis, remove dampness, and promote qi [25]. Shuangshen Decoction contains Morus vulgaris, corn silk, keel, magnet, Polygonum multiflorum, Chuanxiong, Epimedium, and Eucommia. All medicines work together to nourish the kidney and clear away heat [26]. All these results demonstrate that Shuangshen Decoction is beneficial to the treatment of pediatric nephritic syndrome.

In order to improve the curative effect of pediatric nephrotic syndrome and reduce infection and recurrence, this study implemented a comprehensive treatment plan of immune preparations combined with Shuangshen Decoction. Immunosuppressive agents are often used clinically to treat patients with refractory nephropathy or severe hormonal side effects [27]. The dual inhibitory effect of tacrolimus not only makes it able to prevent the occurrence of immunity but also has a good therapeutic effect on the immune response and autoimmune diseases that have appeared [28]. In present study, the overall effect of tacrolimus combined with Shuangshen Decoction was good. Moreover, the recurrence rate and infection rate of patients in the combined group were significantly lower than those in the routine group. The incidence of adverse reactions in the combined group was significantly lower than that in the routine group. These results have not been reported in previous studies. Taken together, Shuangshen Decoction combined with immune preparations are safe and effective in the treatment of pediatric nephrotic syndrome and can also greatly reduce the probability of infection and recurrence.

## 5. Conclusion

In summary, Shuangshen Decoction combined with immune preparations has a significant effect on the treatment of children with nephrotic syndrome. It can increase serum ALB and 24-hour urine protein levels and effectively reduce the incidence of adverse reactions, infection rates, and recurrence rates in children. Due to the small sample size in this study, the sample size will still need to be expanded for further confirmation in the future.

## Figures and Tables

**Figure 1:** The ALB level was compared between the routine group and the combined group. ^∗^*P* < 0.05, ^∗∗^*P* < 0.01.

**Figure 2:** The 24 h urine protein quantification was compared between the routine group and the combined group. ^∗^*P* < 0.05, ^∗∗^*P* < 0.01.

**Figure 3:** The infection rate and recurrence rate were compared between the routine group and the combined group. ^∗^*P* < 0.05, ^∗∗^*P* < 0.01.

**Table 1:** TCM syndrome score sheet (prepared based on relevant information and the clinical experience of the tutor).

Main symptoms	0	2 points	4 points	6 points
Sore waist and knees	None	Occasionally	Frequently	Unbearable
Chills	None	Occasionally	Frequently	Afraid of cold
Poor appetite	None	Reduce food intake by 1/4	Reduce food intake by 1/4-1/2	Little or no food
Secondary symptoms	0	1 point	2 points	3 points
Tired	None	Occasionally	Frequently	Bedridden
Bloating	None	Slightly full	Fullness	Abdominal distension all day
Loose stools	None	1 time/d	2-3 times/d	>4 times/d
Nocturia	None	2 times/night	3 times/night	>4 times/night
Shortness of breath	None	Lack of energy	Lazy in words	Powerless speech
Pale complexion	None	Dull	Pale	Pale and dull

**Table 2:** Comparison of general information between the two groups before treatment.

Index	Routine group (*n* = 45)	Combination group (*n* = 45)	*X* ^2^/*t*	*P*
Age (year)	6.42 ± 1.16	6.55 ± 1.23	0.516	0.607
Course (d)	11.59 ± 2.25	11.68 ± 2.30	0.188	0.852
Gender			0.182	0.670
Male	25 (55.56)	27 (60)		
Female	20 (44.44)	18 (40)		
Disease progression			0.830	0.362
Active nephrotic syndrome	33 (73.33)	29 (64.44)		
Nephrotic syndrome in remission	12 (26.67)	16 (35.56)		
BMI (kg/m^2^)	17.52 ± 2.44	17.69 ± 2.60	0.320	0.750
White blood cell (×10^9^/L)	2.76 ± 0.54	2.85 ± 0.62	0.734	0.465
Cholesterol (mmol/L)	6.88 ± 1.23	6.59 ± 1.17	1.146	0.255
Triglycerides (mmol/L)	3.17 ± 0.84	3.20 ± 0.78	0.176	0.861

**Table 3:** Comparison of TCM syndrome scores between the two groups.

Group	Routine (*n* = 45)	Combination (*n* = 45)	*t*	*P*
Before treatment	15.15 ± 1.20	15.20 ± 1.22		
3 months after treatment	12.47 ± 1.04	9.84 ± 0.72	13.948	<0.001
6 months after treatment	9.91 ± 0.53	7.22 ± 0.41	26.930	<0.001
12 months after treatment	8.84 ± 0.48	4.97 ± 0.51	37.068	<0.001

**Table 4:** Comparison of the clinical efficacy of the two groups [*n* (%)].

Group	Routine (*n* = 45)	Combination (*n* = 45)	*X* ^2^	*P*
Invalid	11 (24.44)	3 (6.67)		
Effective	19 (42.22)	20 (44.44)		
Markedly effective	15 (33.33)	22 (48.89)		
Total effective rate	34 (75.56)	42 (93.33)	5.414	0.020

**Table 5:** Comparison of the incidence of adverse reactions between the two groups [*n* (%)].

Group	Routine (*n* = 45)	Combination (*n* = 45)	*X* ^2^	*P*
Nausea and vomiting	8 (17.78)	2 (4.44)	4.050	0.044
Acne	5 (11.11)	0 (0)	5.294	0.021
Hypertension	6 (13.33)	1 (2.22)	3.873	0.049
Coagulopathy	4 (8.89)	0 (0)	4.186	0.041

## Data Availability

The data used to support the findings of this study are available from the corresponding author upon request.
